# Functional kinomics establishes a critical node of volume-sensitive cation-Cl^−^ cotransporter regulation in the mammalian brain

This article has been retracted.

**DOI:** 10.1038/srep35986

**Published:** 2016-10-26

**Authors:** Jinwei Zhang, Geng Gao, Gulnaz Begum, Jinhua Wang, Arjun R. Khanna, Boris E. Shmukler, Gerrit M. Daubner, Paola de los Heros, Paul Davies, Joby Varghese, Mohammad Iqbal H. Bhuiyan, Jinjing Duan, Jin Zhang, Daniel Duran, Seth L. Alper, Dandan Sun, Stephen J. Elledge, Dario R. Alessi, Kristopher T. Kahle

**Affiliations:** 1 MRC Protein Phosphorylation and Ubiquitylation Unit, College of Life Sciences, University of Dundee, Dundee DD1 5EH, Scotland; 2 Departments of Neurosurgery and Pediatrics, Yale School of Medicine, New Haven, CT 06511 USA; 3 Division of Genetics, Brigham and Women’s Hospital, Boston, MA 02115 USA; 4 Department of Neurology, University of Pittsburgh School of Medicine, Pittsburgh, PA 15213, USA; 5 Department of Cancer Biology, Dana-Farber Cancer Institute, Boston, MA 02115, USA; 6 Department of Biological Chemistry & Molecular Pharmacology, Harvard Medical School, 250 Longwood Ave, SGM 628, Boston, MA 02115, USA; 7 Department of Neurosurgery, Massachusetts General Hospital, Boston, MA 02114 USA; 8 Division of Nephrology and Department of Medicine, Beth Israel Deaconess Medical Center, Boston, MA -022154 USA; 9 Department of Medicine, Harvard Medical School, Boston, MA -022154, USA; 10 Department of Cardiology, Howard Hughes Medical Institute, Boston Children’s Hospital, Boston, Massachusetts 02115, USA; 11 Veterans Affairs Pittsburgh Health Care System, Geriatric Research, Educational and Clinical Center, Pittsburgh, PA, USA; 12 Department of Genetics, Harvard University Medical School, Howard Hughes Medical Institute, Boston, Massachusetts 02115 USA; 13 Departments of Pediatrics and Cellular & Molecular Physiology; Interdepartmental Neuroscience Program; and Centers for Mendelian Genomics, Yale School of Medicine, New Haven, CT 06511 USA

## Abstract

Cell volume homeostasis requires the dynamically regulated transport of ions across the plasmalemma. While the ensemble of ion transport proteins involved in cell volume regulation is well established, the molecular coordinators of their activities remain poorly characterized. We utilized a functional kinomics approach including a kinome-wide siRNA-phosphoproteomic screen, a high-content kinase inhibitor screen, and a kinase trapping-Orbitrap mass spectroscopy screen to systematically identify essential kinase regulators of KCC3 Thr^991^/Thr^1048^ phosphorylation – a key signaling event in cell swelling-induced regulatory volume decrease (RVD). In the mammalian brain, we found the Cl^−^-sensitive WNK3-SPAK kinase complex, required for cell shrinkage-induced regulatory volume decrease (RVI) via the stimulatory phosphorylation of NKCC1 (Thr^203^/Thr^207^/Thr^212^), is also essential for the inhibitory phosphorylation of KCC3 (Thr^991^/Thr^1048^). This is mediated *in vivo* by an interaction between the CCT domain in SPAK and RFXV/I domains in WNK3 and NKCC1/KCC3. Accordingly, genetic or pharmacologic WNK3-SPAK inhibition prevents cell swelling in response to osmotic stress and ameliorates post-ischemic brain swelling through a simultaneous inhibition of NKCC1-mediated Cl^−^ uptake and stimulation of KCC3-mediated Cl^−^ extrusion. We conclude that WNK3-SPAK is an integral component of the long-sought “Cl^−^/volume-sensitive kinase” of the cation-Cl^−^ cotransporters, and functions as a molecular rheostat of cell volume in the mammalian brain.

Vertebrate cells lack rigid cell walls and are highly permeable to water; as such, they face the continuous threat of swelling or shrinkage in response to external or internal osmotic challenges^1^,^2^,^3^. Increases in intracellular osmolality (as occurs in actively-transporting epithelia, metabolically-active cells, or ischemic cells), or decreases in extracellular osmolality (e.g., due to hyponatremia) induce rapid water influx^1^,^4^. The resulting cellular swelling, if unopposed, can rapidly lead to breakdown of cytoskeletal and membrane integrity and subsequent cell death^4^. Even in the absence of osmotic challenge, cells must tightly regulate their volume during cell division, growth, and migration^3^,^5^.

Cell volume regulation involves the rapid adjustment of the activities of plasmalemmal channels and transporters that mediate flux of K^+^, Na^+^, Cl^−^, and small organic osmolytes^3^. This solute transport generates osmotic gradients, which drive water into or out of cells via aquaporin water channels^6^, and perhaps other water-permeant solute transporters^7^. Cell swelling triggers regulatory volume decrease (RVD), which promotes solute and water efflux to restore normal cell volume^4^. Swelling-activated K^+^ and Cl^−^ channels (e.g., volume-regulated anion channel (VRAC), formed by LRRC8 heteromers)^8^,^9^,^10^ and the K^+^-Cl^−^ cotransporters (KCCs, such as KCC3)^11^ mediate RVD in most cell types. In contrast, cell shrinkage triggers regulatory volume increase (RVI), which involves the parallel activation of the Na^+^/H^+^ exchangers NHE1 and Cl^−^/HCO_3_^−^ exchanger AE2, and/or the stimulation of the Na^+^-K^+^-2Cl^−^ cotransporter NKCC1 – a close relative of the KCCs in the cation-Cl^−^ cotransporter family (CCC)^12^. Regulation of RVD and RVI must be tightly coordinated^11^. Whereas the ion transporting “effectors” of RVD and RVI are well characterized, the “sensor” and “transducer” mechanisms that regulate them are less well understood.

The canonical volume-regulated KCCs (KCC1, KCC3, and KCC4) are largely inactive in isotonic conditions, but rapidly activated by cell swelling^13^,^14^,^15^. Swelling-induced KCC activation is abolished by inhibition of protein phosphatase 1A (PP1) and PP2 with calyculin A, demonstrating an essential regulatory role for serine (Ser)-threonine (Thr) kinases/phosphatases in this process^16^,^17^. Conversely, phosphorylation of the KCCs in the setting of cell shrinkage inhibits their activity. Interestingly, the activities of the KCCs and NKCC1 are reciprocally regulated by phosphorylation at structurally homologous Thr residues induced by low intracellular Cl^−^ concentration [Cl^−^]_i_ or hypotonic cell swelling^18^,^19^. In these volume-regulated contexts, protein phosphorylation activates NKCC1 but inhibits KCCs, whereas dephosphorylation produces the reciprocal effects^13^,^14^,^20^,^21^,^22^,^23^. These characteristics have long suggested that the same Cl^−^ and/or volume-sensitive kinase cascade regulates both NKCC1 and the KCCs, but the identities of such molecules has not been systematically examined, nor established *in vivo*.

Two C-terminal Thr residues in human KCC3, Thr^991^ and Thr^1048^, are robustly phosphorylated in isotonic conditions in which the transporter is quiescent, but undergo rapid dephosphorylation in response to cell swelling conditions, which activates the transporter^18^,^19^,^24^. Homologous sites undergo phosphorylation in all human KCCs, including KCC2, and engineered alanine (Ala) substitutions, which prevent phosphorylation at these sites, result in constitutive transporter activity^18^,^19^,^24^. The STE20/SPS1-related proline/alanine-rich kinase (SPAK)^12^,^25^,^26^, known to directly phosphorylate NKCC1 at NKCC1 Thr^203^/Thr^207^/Thr^212^ 27,28, also directly phosphorylates KCC3 Thr^1048^ *in vitro*, but not Thr^991^ 24. However, the molecules that regulate KCC3 Thr^991^/Thr^1048^ phosphorylation *in vitro* have not been systematically examined, or identified *in vivo*. Moreover, the importance of KCC3 Thr^991^/Thr^1048^ phosphorylation for cell volume regulation in the brain remains unknown.

We utilized a functional kinomics approach comprising a kinome-wide siRNA-phosphoproteomic screen, a high-content kinase inhibitor screen, and a kinase trapping-Orbitrap mass spectroscopy screen to systematically identify genes and pathways that regulate KCC3 Thr^991^/Thr^1048^ phosphorylation. The specific goal of our screens was to identify kinases that, when inhibited, would stimulate KCC3 activity by promoting Thr^991^/Thr^1048^ dephosphorylation. Our data converged upon the WNK3-SPAK kinase complex as an essential regulator of KCC3 Thr^991^/Thr^1048^ phosphorylation *in vitro* and *in vivo* in the mammalian brain. Antagonism of WNK3-SPAK signaling was found to facilitate cellular Cl^−^ extrusion by simultaneously decreasing NKCC1 Thr^203^/Thr^207^/Thr^212^ phosphorylation and KCC3 Thr^991^/Thr^1048^ phosphorylation. Accordingly, WNK3-SPAK inhibition prevents acute cell swelling in response to osmotic stress, and ameliorates brain swelling after ischemic stroke. Our data provide evidence that WNK3-SPAK is an integral component of the long-sought “Cl^−^/volume-sensitive kinase” of the cation-Cl^−^ cotransporters, and functions as a molecular rheostat of cell volume in the mammalian brain.

## Results

### An RNAi screen for kinases essential for KCC3 Thr^991^ phosphorylation

We carried out a kinome-wide RNAi screen in human HEK293 cells with doxycycline (dox)-inducible expression of MYC-tagged human KCC3^18^,^19^ to identify genes required for KCC3 Thr^991^ phosphorylation (herein “KCC3 P-Thr^991^”). We employed a phospho-specific antibody that recognizes KCC3 P-Thr^991^ as a reporter for the screen^24^. We reasoned that kinases regulating KCC3 P-Thr^991^ might also regulate P-Thr^1048^, since the phosphorylation of these sites are induced by the same stimuli with similar kinetics^19^. The signal of KCC3 P-Thr^991^ antibody is robust in isotonic conditions, inversely correlates with the activity of KCC3, and is significantly decreased in response to hypotonic cell swelling conditions that stimulate KCC3 activity, or when Thr^991^ is mutated to alanine (Ala) to prevent phosphorylation^18^,^19^ (Fig. 1A,B).

In the primary screen of HEK293-KCC3 cells, we depleted individual proteins using the human Dharmacon SMARTpool siRNA kinome library, which targets 720 kinases and associated proteins, including nearly all serine, threonine, tyrosine, and lipid kinases, using pools of 4 independent siRNA oligonucleotides target different regions of each gene. Knockdown by each siRNA was performed in triplicate in 24-well plates. After induction of MYC-KCC3 expression by dox in siRNA-transfected cells, we harvested cell lysates and subjected them to SDS-PAGE gel fractionation and Western blot analysis with anti-KCC3 P-Thr^991^ antibody^24^. The KCC3 P-Thr^991^ immuno-signal on Western blots was quantitated as described in Methods (Fig. 1C).

Negative control firefly (FF) luciferase siRNAs had no effect on KCC3 P-Thr^991^; in contrast, positive control siRNAs targeting KCC3 itself knocked down the KCC3 P-Thr^991^ signal almost entirely. The primary screen resulted in the identification of multiple siRNA pools that led to a consistent and significant (>50%, p < 0.01) *decrease* in KCC3 P-Thr^991^ signal. We performed robust z-score analysis^29^ of the data from the primary screen (Fig. 1D), and candidates with highly negative z-scores (i.e., siRNAs that decreased the KCC3 P-Thr^991^ immuno-signal more than two standard deviations below the mean of the buffer-alone and the negative control FF siRNAs) These hits included serine-threonine kinases, tyrosine kinases, and lipid kinases (*ITPKC*, *AKT1*, *FRAP1*, *EPHA10*, *DGKK*, *PRKCM*, *CIB2*, *PRKWNK3*, *MATK*, *HRI*, *PI4K2B*, *ROR1*, *TGFBR3*, *LOC390226*, *NME2*, *JIK*, *ROCK2*, *SGK1*, *MYLK*, and *AK2*), and were considered for further analysis by a secondary screen.

The secondary screen analyzed siRNAs targeting the above candidates for their ability to specifically decrease KCC3 P-Thr^991^ without altering total KCC3 protein expression, as detected by anti-MYC antibody. For each candidate siRNA pool, we calculated the ratio of anti-KCC3 P-Thr^991^ and anti-MYC immunoblot signals. Given that KCC3 Thr^991^ is strongly phosphorylated in isotonic conditions, this ratio for negative control FF luciferase siRNA was normalized to 1. Thirteen genes yielded significantly decreased “KCC3 P-Thr^991^-to-MYC” ratios, including *EPHA10*, *PRKCM*, *JIK*, *ROR1*, *ROCK2*, *CIB2*, *MATK*, *AK2*, *WNK3*, *AKT1*, *PI4K2B*, *SGK1*, and *DGKK*; Fig. 1E). Analysis of these hits using the Search Tool for the Retrieval of Interacting Genes/Proteins (STRING) database revealed several protein-protein interactions (http://string-db.org), including clusters of kinases known to participate in the regulation of ion transport, cell volume regulation, and cell size (Fig. 1F).

These targets were further validated and siRNA off-target signals minimized^30^ by employing a tertiary screen that investigated the effects of genomic knockout (KO) of candidate kinases on KCC3 P-Thr^991^ in cell lines (see Methods). This strategy allowed validation of our findings in other cell types, including mouse embryonic fibroblasts (MEFs) and mouse embryonic stem cells (mESCs). To identify kinases that might *directly* phosphorylate KCC3, we limited the tertiary (validation) screen to only serine-threonine kinases. We examined KCC3 P-Thr^991^ using phospho-antibodies in cell lines knocked out for WNK3, PRKD1 (i.e., encoding Protein Kinase D1 [PKD1], also known as PKC-Mu), AKT1, ROCK2, and TSC1 and TSC2 (as models harboring significantly decreased AKT1 and SGK1 activity^31^,^32^,^33^,^34^. KCC3 P-Thr^1048^ and NKCC1 P-Thr^203^/Thr^207^/Thr^212^ were also monitored with phospho-antibodies^24^,^28^ (Fig. 1A). In hypotonic low Cl^−^ conditions, NKCC1 activity is stimulated via phosphorylation at Thr^203^/Thr^207^/Thr^212^; in the same conditions, KCC3 activity is inhibited due to phosphorylation at Thr^991^/Thr^1048^ 24,28. KCC3 Thr^991^ and NKCC1 Thr^212^ are located in highly homologous sequence contexts, suggesting a common phospho-motif^19^.

In conditions promoting CCC phosphorylation, WNK3 KO cells exhibited apparently decreased levels of KCC3 P-Thr^991^ (>1.5-fold, *p* < *0.01*), KCC3 P-Thr^1048^ (>1.4-fold, *p* < *0.05*), and NKCC1 P-Thr^203^/Thr^207^/Thr^212^ (>1.4-fold, *p* < *0.01*) (Fig. 2A and Supplementary Figure 1A). PKD1 KO cells also exhibited decreases of KCC3 P-Thr^991^ (>2 fold, *p* < *0.001*), P-Thr^1048^ (>1.8, *p* < *0.01*) and NKCC1 P-Thr^203^/Thr^207^/Thr^212^ (>1.4 fold, *p* < *0.05*) (Fig. 2B and Supplementary Figure 2A). In contrast, AKT1 KO and ROCK2 KO cells exhibited no apparent change in either KCC3 P-Thr^991^/Thr^1048^ or NKCC1 P-Thr^203^/Thr^207^/Thr^212^. Moreover, TSC1 KO and TSC2 KO cells (containing *reduced* levels of activated AKT1 and SGK1^31^,^32^,^33^,^34^, showed apparently *increased* levels of KCC3 P-Thr^991^/Thr^1048^ (>1.3-2 fold, *p* < *0.05*; Fig. 2C and Supplementary Figure 2B). These data show WNK3 and PDK1, but not AKT1, SGK1, or ROCK2, are essential for KCC3 P-Thr^991^/Thr^1048^ and NKCC1 P-Thr^203^/Thr^207^/Thr^212^.

### A screen to identify kinase inhibitors that antagonize KCC3 Thr^991^/Thr^1048^ phosphorylation

To corroborate and extend findings from our RNAi screen, we performed a high content drug screen of a library containing >220 well-characterized, cell-permeable protein kinase inhibitors to identify individual kinases or signaling pathways required for phosphorylation of KCC3 Thr^991^/Thr^1048^ (Fig. 3A; see Methods for details).

In the primary screen, dox-induced HEK293 KCC3 cells were exposed to 20 μM kinase inhibitor for 2 hours in 24-well plates, followed by lysate harvest, gel fractionation, and semi-quantitative Western blot analysis of KCC3 P-Thr^991^ and total KCC3 protein. Negative control DMSO had no effect on KCC3 P-Thr^991^; in contrast, positive controls Torin 1 and Rapamycin robustly decreased pS6K P-Thr^389^. Of 220 kinase inhibitors tested, 32 different drugs significantly decreased KCC3 P-Thr^991^ when assayed at 20 μM for 2 hours in isotonic conditions (Fig. 3A). These hits included the WNK-SPAK kinase CCT domain inhibitor STOCK1S-50699 35; multiple drugs targeting the PI3K-AKT-mTOR pathway, including GDC-0941, ZSTK474, AS605240, and AZD-6482 (PI3K); KIN001-102, MK2206, and SB590885 (AKT), and Rapamycin, AZD8055, PP242, and Torin1/2 (mTOR); and several drugs targeting MAPK-associated pathways including HER2 (CP724714, HKI-272, and GW-572016); PLK1 (GSK461364, GW843682, and BI-2536); B-Raf (PLX4032 and PLX-4720); and p38 (TAK-715 and SB 239063) (Fig. 3A).

In the secondary drug screen, we tested representative positive primary screen candidates of specific pathways at lower concentrations and with decreased incubation times to promote increased drug specificity (1 μM for 30 min; see Methods). We assessed the effects of drugs on *endogenous* KCC3 P-Thr^991^ to avoid non-specific effects of protein over-expression. We also tested drugs in the presence or absence of hypotonic, low Cl^−^ conditions to select for phosphorylation events specific for cell volume homeostasis^24^. Of all kinase inhibitors tested in the secondary screen, only STOCK1S-50699 substantially decreased KCC3 P-Thr^1048^ (Fig. 3B). In addition, STOCK1S-50699 was the only compound that substantially decreased NKCC1 P-Thr^203^/Thr^207^/Thr^212^ (Fig. 3C).

We characterized the effect of STOCK1S-50699 on SPAK P-Ser^373^, KCC3 P-Thr^991^/Thr^1048^, and NKCC1 P-Thr^203^/Thr^207^/Thr^212^ in dose-response experiments (Fig. 3C,D). STOCK1S-50699 showed a graded inhibitory effect on SPAK P-Ser^373^, consistent with SPAK inhibition (Fig. 3C,D)^24^. STOCK1S-50699 also had a graded inhibitory effect on KCC3 P-Thr^991^ with doses between 3–10 μM in activating conditions. In contrast, STOCK1S-50699 treatment eliminated KCC3 P-Thr^1048^ and NKCC1 P-Thr^203^/Thr^207^/Thr^212^ even when tested at a concentration of 1 μM (Fig. 3C,D). These data show STOCK1S-50699 simultaneously inhibits KCC3 P-Thr^1048^ and, with less potency, KCC3 P-Thr^991^, as well as NKCC1 P-Thr^203^/Thr^207^/Thr^212^. These results also show KCC3 Thr^991^/Thr^1048^ phosphorylation is a specific event, not affected by a panel of common kinase inhibitors, when tested at physiologically relevant doses and short incubation times.

### Kinase trapping-Orbitrap mass spectroscopy to identify kinase regulators of KCC3

Proteins responsible for KCC3 Thr^991^/Thr^1048^ phosphorylation might differentially bind to the KCC3 C-terminus depending on transporter exposure to activating (dephosphorylating) cell swelling conditions, or inhibitory (phosphorylating) isotonic control conditions. To identify protein kinases that interact with and potentially regulate KCC3 P-Thr^991^/Thr^1048^, we performed kinase trapping coupled with Orbitrap MS^36^; see Methods for details).

Briefly, HEK293 cells expressing FLAG-tagged KCC3 were exposed to either control isotonic buffer (KCC3 P-Thr^991^/Thr^1048^) or cell swelling hypotonic buffer (KCC3 deP-Thr^991^/Thr^1048^). Lysates incubated with or without phosphatase inhibitors were purified by affinity chromatography in two separate columns, to “trap” KCC3 phospho-regulatory elements. Both KCC3 P-Thr^991^/Thr^1048^and (de)P-Thr^991^/Thr^1048^ were immunoprecipitated by FLAG antibody and analyzed by Orbitrap MS.

Only several different kinases were found to associate with the phosphorylated and/or dephosphorylated species of KCC3. SPAK, microtubule associated serine/threonine kinase-like (MASTL), the serine/threonine-protein kinase tousled-like 2 (TLK2), and mTOR interacted with both phosphorylated and de-phosphorylated KCC3 with very high Mascot scores (Table 1). The SPAK ortholog OSR1 and phosphoglycerate kinase 1 (PGK1) selectively interacted with only the dephosphorylated KCC3.

We assessed whether identified candidate kinases from our screens *directly* phosphorylated KCC3. We tested whether purified (and active) SPAK, WNK3, WNK1 (an ortholog of WNK3), PDK1, SGK1, or TLK2, directly phosphorylate the KCC3 N-terminus (aa 1–175) or C-terminus (aa 886–1141, containing Thr^991^ and Thr^1048^) in *in vitro* kinase assays (Supplementary Figure 3). SPAK, in the presence or absence of its regulatory MO25α subunit^37^, phosphorylated KCC3 Thr^1048^ but not KCC3 Thr^991^ 24. In contrast, WNK3, WNK1, PDK1, TLK2, or SGK1 did not result in phosphorylation of the KCC3 N-terminus, or the C-terminus encompassing Thr^991^ and Thr^1048^ (Supplementary Figure 3). These results demonstrate SPAK directly phosphorylates KCC3 Thr^1048^ but not Thr^991^, and that WNK3 and PDK1, while essential for full KCC3 Thr^991^ and Thr^1048^ phosphorylation, likely indirectly regulate these sites.

### WNK3 inhibition facilitates KCC3-dependent Cl^−^ extrusion by decreasing Thr^991^ and Thr^1048^ phosphorylation

We analyzed endogenous KCC3 activity in WNK3 wild type (WT) and WNK3 KO mES cells by measuring ^86^Rb^+^ uptake in isotonic control conditions, hypotonic high K^+^ conditions (KCC3 Thr^991^/Thr^1048^ dephosphorylated and active), and hypotonic low Cl^−^ conditions (KCC3 Thr^991^/Thr^1048^ phosphorylated and inactive) (see Methods; Fig. 4A and Supplementary Figure 1A and Supplementary Figure 4A). Exposure of WT WNK3 cells to hypotonic high K^+^ conditions activated ^86^Rb^+^ uptake by ~1.5-fold^24^. WNK3 mES KO cells displayed a significantly increased level of basal ^86^Rb^+^ uptake in isotonic control conditions that was further stimulated by hypotonic high K^+^ conditions (p < 0.001), but not hypotonic low Cl^−^ conditions. These results are consistent with increased KCC3 activity secondary to Thr^991^/Thr^1048^ dephosphorylation (Supplementary Figure 4A).

We next examined activities of WT KCC3, KCC3^Thr991Ala^, and KCC3^Thr1048Ala^ in HEK293T WT, WNK1 KO and WNK3 KO cells (generated by Crispr/CAS9) by measuring ^86^Rb^+^ uptake in control isotonic and hypotonic low Cl^−^ conditions (Fig. 4B). Under hypotonic low Cl^−^ conditions, both WNK1 KO cells and WNK3 KO cells showed *decreased* phosphorylation of both endogenous and heterologously-expressed KCC3 at Thr^991^ (*p* < *0.001*) and Thr^1048^ (*p* < *0.001*). HEK293T WNK1 KO cells and WNK3 KO cells also showed apparently *decreased* NKCC1 P-Thr^203^/Thr^207^/Thr^212^, SPAK P-Ser^373^, and OSR1 P-Ser^325^ (*p* < *0.05 for each*; Fig. 4D,E, Supplementary Figure 4D,E). Individual mutation of either KCC3 Thr^991^ or Thr^1048^ to Ala apparently activated KCC3, and each single mutant was apparently further stimulated by hypotonic low Cl^−^ conditions or by hypotonic high K^+^ conditions in both WNK1-KO (*p* < *0.05*) and WNK3-KO cells (*p* < *0.05*) (Fig. 4B). STOCK1S-50699 treatment of cells expressing KCC3^Thr991Ala^, KCC3^Thr1048Ala^ or the double mutant KCC3^Thr991Ala/Thr1048Ala^ did not change KCC3 activity, suggesting that Ala mutation of these Thr residues abolishes WNK3-SPAK-mediated inhibitory phosphorylation (Fig. 4C and Supplementary Figure 4C). These results together suggest that WNK3 inhibition facilitates KCC3-dependent Cl^−^ extrusion by decreasing KCC3 P-Thr^991^/Thr^1048^.

### WNK3-SPAK inhibition prevents acute cell swelling by stimulating KCC3 activity

The importance of KCC3 P-Thr^991^ and P-Thr^1048^ in RVD^18^,^19^ prompted the speculation that WNK3-SPAK inhibition might alter the acute cell swelling response induced by osmotic stimuli. We therefore assessed the relative change in cell water content to acute hypotonic swelling in HEK293 cells (see Methods) expressing WT WNK3 or kinase-dead (KD) WNK3 in the presence or absence of STOCK1S-50699 (Fig. 5). Stimulation of WNK3-WT cells with hypotonic HEPES-MEM (150 mOsm/kg H_2_O) swelled cells ~3 ± 0.2-fold in volume (Fig. 5A), whereas WNK3-KD cells swelled only 1.2 ± 0.1-fold (, p < 0.05). Hypotonically-stressed WNK3-WT cells swelled at 1.03 ± 0.1% cell volume/min (Fig. 5A), whereas WNK3-KD cells swelled at only 0.4 ± 0.1% cell volume/min. Exposure of WNK3-WT cells to STOCK1S-50699 prevented cells from swelling in response to acute hypotonic stress (Fig. 5B). WNK3-KD cells treated with STOCK1S-50699 showed no additional reduction in cell swelling (Fig. 5C). Treatment of cells with 2 mM furosemide, which at this concentration inhibits KCC3, abrogated the effect of WNK3-KD on hypotonic cell swelling (Fig. 5D). These results demonstrate WNK3-SPAK inhibition prevents acute cell swelling in response to osmotic stress by stimulating KCC3 activity.

### A WNK3/SPAK complex regulates NKCC1/KCC3 phosphorylation in the ischemic brain

In the mammalian brain, glia outnumber neurons and significantly contribute to total brain volume. Unlike neurons, glia express aquaporin water channels, rendering them more sensitive to osmotic perturbation^11^. As such, impaired glial cell volume homeostasis disproportionately contributes to the cerebral edema^11^. NKCC1 and KCC3 are highly expressed in astrocytes and endothelial cells of the blood-brain-barrier (BBB)^38^,^39^. Brain ischemia, as modeled experimentally by middle cerebral artery occlusion (MCAO), causes the NKCC1-dependent cytotoxic edema of astrocytes^38^,^40^ and BBB endothelial cells^41^,^42^,^43^. These collectively contribute to BBB breakdown, vasogenic edema, and brain swelling^44^,^45^. WNK3 KO mice develop significantly less cerebral edema and infarct volume after MCAO, and exhibit accelerated neurobehavioral recovery, but the mechanisms of these effects remain incompletely understood^46^.

We examined KCC3 P-Thr^991^/Thr^1048^ and NKCC1 P-Thr^203^/Thr^207^/Thr^212^ in WNK3 WT and KO mice post-MCAO using phospho-specific antibodies (Fig. 6A). At 6 and 24 hours post-MCAO, WNK3 KO mice exhibited a 2.0–2.5-fold apparent decrease in NKCC1 P-Thr^203^/Thr^207^/Thr^212^ (*p* < *0.01*) and a 2.0–2.7-fold apparent decrease in KCC3 P-Thr^1048^ (*p* < *0.05*; Fig. 6A) compared to WNK3 WT mice. SPAK CCT domain knock-in mice (*SPAK*^*502A*^*/*^*502A*^) harbor a genetic mutation that inhibits *in vivo* WNK kinase-dependent SPAK kinase activation^47^. This mutation disrupts a physical interaction between the RFXV/I motifs of WNKs and CCCs with the conserved carboxyl-terminal (CTT) docking domain in SPAK^47^, thus genetically mimicking the effect of STOCK1S-50699^35^. We examined KCC3 P-Thr^991^/Thr^1048^ and NKCC1 P-Thr^203^/Thr^207^/Thr^212^ in WT and *SPAK*^*502A/502A*^ mice using phospho-specific antibodies (Fig. 6C,D).

Similar to WNK3 KO mice, *SPAK*^*502A/502A*^ mice exhibited an apparent 2.5~3.0-fold decrease in NKCC1 P-Thr^203^/Thr^207^/Thr^212^ (*p* < *0.01*) and KCC3 P-Thr^1048^ (*p* < *0.001*) (Fig. 6C,D). Moreover, *SPAK*^*502A/502A*^ mice also exhibited an apparent 2.5~3.0-fold decrease in KCC2 P-Thr^906^/Thr^1007^ (*p < 0.01*), sites homologous to KCC3 Thr^991^/Thr^1048^ (Fig. 6C,D).

We also tested the physical interaction of WNK3 and SPAK with KCC3 in the brain. Reciprocal co-immunoprecipitation experiments revealed that both WNK3 and SPAK formed a complex with KCC3 in WT mouse brain, but not in littermate WNK3 KO brains, or in KCC1/3 double KO brains^48^,^49^ (Fig. 6E). In addition, co-immunoprecipitation of KCC3 with SPAK was abrogated in *SPAK*^*502A*^*/*^*502A*^ mice (Fig. 6C). Together, these data show that NKCC1 and KCC3 phosphorylation in the brain is regulated by a WNK3-SPAK complex and mediated in part by an interaction between the CCT in SPAK and RFXV/I domains in WNK3 and NKCC1/KCC3.

### WNK3/SPAK inhibition decreases the cytotoxic edema of astrocytes and endothelial cells of the blood-brain barrier

Ischemia-induced cytotoxic swelling of astrocytes is associated with reactive gliosis marked by hypertrophy, proliferation, and up-regulation of the astrocyte-specific marker glial fibrillary acidic protein (GFAP) and AQP4 located at peri-capillary astrocytic end feet^50^. We assessed the ischemia-induced cytotoxic swelling of astrocytes after MCAO in WNK3 WT and WNK3 KO mice. MCAO triggered astrocyte hypertrophy in the ipsilateral ischemic peri-infarct cortex of WNK3 WT brains, as evidenced by increased soma volume of stellate astrocytes (defined by GFAP staining (GFAP^+^) that harbor multiple enlarged radiating processes (Arrows; Fig. 6F). In contrast, the number and soma volume of GFAP+ astrocytes were significantly reduced in WNK3 KO brains after MCAO (*p* < *0.05*, WT vs. KO, Fig. 6F).

Ischemia-induced cytotoxic swelling of BBB endothelial cells and astrocytic end feet disrupts BBB integrity and causes vasogenic cerebral edema^51^,^52^,^53^. We detected less reactive astrocyte formation at AQP4-stained end feet associated with BBB endothelial cells in post-MCAO WNK3 KO brains than in WNK3 WT brains. Since systemic IgG does not cross the BBB^54^, we investigated BBB integrity in WNK3 WT and WNK3 KO brains by measuring IgG infiltration^55^. Increased BBB permeability was detected in WNK3 WT mice 3 days after ischemic stroke, as reflected by greatly increased IgG accumulation in ipsilateral peri-lesional cortices (Fig. 6G; *p* < *0.05*). In contrast, WNK3 KO brains exhibited significantly less IgG infiltration (Fig. 6G; *p* < *0.05*). These results demonstrate that WNK3 KO reduces BBB breakdown associated with endothelial cell cytotoxic swelling.

## Discussion

We have identified the regulatory elements controlling phosphorylation of KCC3 at residues Thr^991^ and Thr^1048^, a key signaling event of the homeostatic response to cell swelling that triggers RVD^19^,^24^. Our multi-tiered functional kinomics approach included a kinome-wide siRNA-phosphoproteomic screen, a high-content kinase inhibitor drug screen, and kinase trapping coupled with Orbitrap MS. We used multiple, complementary screening and validation assays to improve chances for unbiased detection of important and possibly novel regulatory elements while minimizing “off-target” effects. For example, to improve screen specificity we validated siRNA screen hits not with other siRNAs, but with KO cell lines. Complementation of the siRNA loss-of-function kinome screen with a kinase inhibitor drug screen allowed assessment of kinase inhibition effects in different cell types on different time scales. The ability of kinases to regulate transporter phosphorylation was assayed both indirectly (with anti-phospho antibodies) and directly (using *in vitro* kinase assays). Moreover, we validated *in vitro* findings using the *in vivo* brain MCAO *in vivo* model of ischemic cerebral edema.

Collectively, our results converged on the WNK-SPAK kinase as a particularly important node of KCC3 P-Thr^991^/Thr^1048^ phosphorylation. Components of this pathway were represented in all 3 types of screens: 1) *WNK3* was identified in the siRNA screen, and validated in KO cell lines (Figs 1, 2, 3, 4 and 5); STOCK1S-50699, which inhibits SPAK activation by the WNK kinases, including WNK3, was identified in the kinase inhibitor screen and validated with dose-response and functional experiments (Fig. 3); SPAK and its homolog OSR1 was identified in kinase Orbitrap MS experiments (Table 1). In addition, both WNK3 and SPAK were validated *in vivo* in brain (Fig. 6). Among the >200 kinase inhibitors tested at the concentrations recommended to achieve target specificity, STOCK1S-50699 was unique in targeting KCC3 P-Thr^991^ and P-Thr^1048^. Our experiments reveal a hitherto unrecognized specificity of regulation of KCC3 P-Thr^991^/Thr^1048^ by the WNK-SPAK kinase pathway, and show for the first time the requirement of these kinases for KCC3 phosphorylation *in vivo*. Further experiments revealed additional novel insights into this pathway: while SPAK directly phosphorylates Thr^1048^, it does not phosphorylate Thr^991^ (Fig. 6C,D). Also, while WNK3 is required for both P-Thr^991^ and P-Thr^1048^, it does not appear to phosphorylate either residue directly, as shown by *in vitro* kinase assays (Supplementary Figure 3A). Moreover, although STOCK1S-50699 inhibits both KCC3 P-Thr^991^ and P-Thr^1048^, the drug more potently inhibits P-Thr^1048^ at lower concentrations (Fig. 3C).

Our *in vivo* validation experiments with WNK3 and SPAK uncovered novel insights into the roles of this swelling-regulated pathway in the mammalian brain. We showed these kinases interact *in vivo* in brain, and that genetic knockdown of WNK3, or prevention of SPAK activation by the WNKs via missense mutation in the CCT domain of SPAK (*SPAK*^*502A/502A*^), each decreases KCC3 P-Thr^1048^ and, to a lesser extent, KCC3 P-Thr^991^. Genetic inhibition of WNK3-SPAK signaling in the MCAO model also ameliorated two cell swelling-associated components of ischemic cerebral edema: perivascular cytotoxic edema of astrocytes and endothelial cell cytotoxic edema (both contributing to BBB breakdown). These findings provide a mechanistic explanation for the improved radiographic and clinical outcomes of malignant cerebral edema after ischemic stroke in mice genetically lacking either WNK3 or SPAK^46^. Our *in vitro* data (Fig. 6) suggest that this *in vivo* effect likely results from increased KCC3-dependent cellular Cl^−^ efflux due to decreased inhibitory KCC3 phosphorylation.

We hypothesized that any kinases shown to regulate KCC3 P-Thr^991^ and/or P-Thr^1048^ might also regulate NKCC1 at a homologous phosphorylation motif (Thr^203^/Thr^207^/Thr^212^) by the same stimuli, but with reciprocal effects^12^,^24^. Indeed, our *in vitro* and *in vivo* data show that WNK3-SPAK signaling is required for the simultaneous volume-regulated phosphorylation of both KCC3 and NKCC1 in our cell culture systems and in the ischemic brain. The existence of a common Cl^−^/volume sensitive regulatory kinase that reciprocally regulates both the NKCCs and the KCCs has long been proposed^16^, but experimental evidence for these simultaneous effects in the same mammalian cells *in vitro* or *in vivo* has been lacking. We show here that knockout of WNK3 in cells, blockade with STOCK1S-50699, or genetic inactivation of the WNK3-SPAK kinase pathway in the brain (in the setting of ischemic conditions promoting cell swelling) simultaneously antagonizes inhibitory KCC3 P-Thr^991^/Thr^1048^ and stimulatory NKCC1 P-Thr^203^/Thr^207^/Thr^212^. These inhibitory effects are predicted to facilitate net Cl^−^ extrusion from cells by concurrent inhibition of Cl^−^ loading by NKCC1 and stimulation of Cl^−^ efflux by KCC3, and can explain the decreased cerebral edema observed post-MCAO in WNK3 KO mice^56^.

Our screens also identified several novel candidate regulators of KCC3 such as PDK1 kinase (Fig. 1B–E and Supplementary Figure 2A). *In vitro* kinase assays suggest that PDK1 does not directly phosphorylate KCC3, but could perhaps mediate its effect via another kinase, similar to the action of WNK3. TLK2 and other novel kinases were also found to interact with phospho- or dephospho-KCC3, although TLK2 did not phosphorylate KCC3 directly. Both primary siRNA and drug screens identified multiple kinases in the mTOR pathway, including SGK1 and AKT1. However, validation of these targets failed in KO cell lines or when drugs were used at lower concentrations to achieve higher target specificity. Notably, the mTOR-AKT1-SGK1 pathway has been previously implicated in regulation of the WNK-SPAK signaling pathway^57^,^58^. Thus, *transient* inhibition of multiple isoforms of mTOR pathway components such as SGK or AKT, might regulate KCC3/NKCC1 phosphorylation via mechanisms independent of or dependent on the WNK-SPAK pathway, whereas selective inhibition of single isoforms (e.g., SGK1 or AKT1), or constitutive inhibition by genetic knockout might allow or stimulate counter-regulatory pathways. The known roles of the mTOR-AKT1-SGK1 pathway in regulation of cell size and volume suggest a possible swelling-independent mechanism involving KCC3. These observations emphasize the need for further investigation of these novel kinase hits in future experiments.

These results suggest a model that links the Cl^−^/volume-sensitive WNK3-SPAK kinase complex with both NKCC1 and KCC3 to comprise a “molecular rheostat” of cell volume homeostasis, balancing opposing, phosphorylation-mediated effects on these two transporters (Fig. 7). The existence of such a kinase system has been proposed^59^, but its molecular identity has not systematically studied or characterized *in vivo*. We suggest that the WNK3-SPAK complex serves as a combined “sensor-transducer” that simultaneously signals both to the RVI effector, NKCC1 and to the RVD effector KCC3. Interestingly, both WNK3 and NKCC1/KCC3 contain RFXV/I motifs, which mediate docking with the conserved C-terminal (CCT) domain of SPAK^60^. This interaction appears unique in the genome, and therefore constitutes a compelling drug target. As such, our results documenting beneficial effects of WNK3-SPAK inhibition in the MCAO model of cerebral edema suggest this complex could be as a novel therapeutic target for a medical problem of high morbidity and mortality commonly associated with stroke, tumor, trauma, infection, and other intracranial pathologies^61^. Given the finding that SPAK inhibition also simultaneously decreases KCC2 P-Thr^1007^ (see Fig. 6C), a site homologous to KCC3 P-Thr^1048^ that, when dephosphorylated, potentiates neuronal Cl^−^ extrusion^24^, we speculate that neuronal WNK-SPAK inhibition could be a potential novel strategy to restore GABA inhibition in hyper-excitable neurons with high intracellular [Cl^−^]. Taken together, our study provides comprehensive evidence for the WNK3/SPAK-mediated regulation of KCC3 and NKCC1 protein phosphorylation and function in cell volume homeostasis.

## Methods

### Kinome siRNA-phosphoproteomic screen

To identify genes required for KCC3 P-Thr^991^ phosphorylation, a high-throughput RNAi screen was performed in 24-well plates with the human Dharmacon SMARTpool siRNA kinome library targeting 541 kinases and kinase-related genes in which each mRNA is targeted by a pool of siRNAs consisting of a combination of four siRNA duplexes directed at different regions of the gene. This siRNA library has been previously characterized and extensively used^62^,^63^,^64^,^65^,^66^,^67^. The HEK293 cell line with Flip-in TREX dox-inducible expression of MYC-tagged KCC3 18,19 was seeded in 24-well plates at the density of 2.5 × 10^6^ cells per well. Each well of cells was transfected with 100 nM of siRNA pool containing 25nM of each of four siRNAs targeting each gene, using by Mirus TransIT TKO reagent. Additional wells present on all plates transfected contained either buffer alone, a non-targeting control siRNA (siGENOME non-targeting siRNA #2, Dharmacon, or firefly (FF) luciferase), and siRNAs directed against KCC3^19^. After 48 hours of culture and dox-induction of MYC-KCC3 expression in siRNA-transfected cells as described^18^, we harvested membrane lysates and subjected them to SDS-PAGE gel fractionation and Western blot analysis with anti-KCC3 P-Thr^991^ antibody. The level of the KCC3 P-Thr^991^ immuno-signal on Western blots was quantitated using ImageJ software, and robust z-score analysis^29^ of the primary screen data was performed. siRNAs that decreased KCC3 P-Thr^991^ immuno-signal >2 SD below the mean of the buffer-alone and negative control wells were considered as identifying candidate kinases for further investigation.

### Antibodies

The following antibodies were raised in sheep and affinity-purified on the appropriate antigen by the Division of Signal Transduction Therapy Unit at the University of Dundee: KCC2 total antibody [S700C, first bleed; raised against residues 1–119 of human KCC2A]; KCC3 total antibody [S701C, first bleed; raised against residues 1–175 of human KCC3]; KCC3 phospho-Ser^96^ antibody [S042D, first bleed; raised against residues 89–103 of human KCC3 phosphorylated at Ser^96^, IEDLSQN(S)ITGEHSQ]; KCC3 phospho-Thr^991^ [S959C, first bleed; raised against residues 984–998 of human KCC3A phosphorylated at Thr 991, SAYTYER(T)LMMEQRSRR]; KCC3 phospho-Thr^1048^ [S961C, first bleed; raised against residues 1041–1055 of human KCC3 phosphorylated at Thr^1048^, CYQEKVHMT*WTKDKYM]. NKCC1 total antibody [S022D, second bleed; raised against residues 1–288 of human NKCC1]; NKCC1 phospho-Thr^203^/Thr^207^/Thr^212^ antibody [S763B, third bleed; raised against residues 198–217 of human NKCC1 phosphorylated at Thr^203^, Thr^207^ and Thr^212^, HYYYD(T)HTN(T)YYLR(T)FGHNT]; WNK1-total antibody [S079B, second bleed; raised against residues 2360–2382 of human WNK1]; WNK1-phospho-Ser^382^ antibody [S099B, second bleed; raised against residues 377–387 of human WNK1 phosphorylated at Ser^382^, ASFAK(S)VIGTP]; WNK2-total antibody [S140C, second bleed; raised against residues 1605–1871 of human WNK2]; WNK3-total antibody [S156C, second bleed; raised against residues 1142–1461 of human WNK3]; WNK4-total antibody [S064B, second bleed; raised against residues 1221–1243 of human WNK4]; SPAK-total antibody [S551D, third bleed; raised against full-length GST-tagged human SPAK protein]; SPAK-N termial antibody [S668D, third bleed; raised against residues 2–76 of mouse SPAK]; SPAK/OSR1 (S-motif) phospho-Ser^373^/Ser^325^ antibody [S670B, second bleed; raised against residues 367–379 of human SPAK, RRVPGS(S)GHLHKT, which is highly similar to residues 319–331 of human OSR1 in which the sequence is RRVPGS(S)GRLHKT); ERK1 total antibody [S221B, second bleed; raised against full-length human ERK1 protein]. The anti-FLAG antibody (F1804) was purchased from Sigma-Aldrich; the anti-PDK1 antibody (3062) and the Tuberin/TSC2 (28A7) antibody (3635) were purchased from Cell Signaling Technology. Secondary antibodies coupled to horseradish peroxidase used for immunoblotting were obtained from Pierce. IgG used in control immunoprecipitation experiments was affinity-purified from pre-immune serum using Protein G-Sepharose.

### Buffers

Buffer A contained 50 mM Tris/HCl, pH7.5 and 0.1 mM EGTA. Lysis buffer was 50 mM Tris/HCl, pH 7.5, 1 mM EGTA, 1 mM EDTA, 50 mM sodium fluoride, 5 mM sodium pyrophosphate, 1 mM sodium orthovanadate, 1% (w/v) NP-40, 0.27 M sucrose, 0.1% (v/v) 2-mercaptoethanol and protease inhibitors (1 tablet per 50 ml). TBS-Tween buffer (TTBS) was Tris/HCl, pH 7.5, 0.15 M NaCl and 0.2% (v/v) Tween-20. SDS sample buffer was 1X-NuPAGE lithium dodecyl sulfate (LDS) sample buffer (Invitrogen), containing 1% (v/v) 2-mercaptoethanol. Isotonic high potassium buffer was 95 mM NaCl, 50 mM KCl, 1 mM CaCl_2_, 1 mM MgCl_2_, 1 mM Na_2_HPO_4_, 1 mM Na_2_SO_4_ and 20 mM HEPES (pH 7.4). Hypotonic high potassium buffer was 80 mM KCl, 1 mM CaCl_2_, 1 mM MgCl_2_, 1 mM Na_2_HPO_4_, 1 mM Na_2_SO_4_ and 20 mM HEPES (pH 7.4). Isotonic buffer was 135 mM NaCl, 5 mM KCl, 0.5 mM CaCl_2_, 0.5 mM MgCl_2_, 0.5 mM Na_2_HPO_4_, 0.5 mM Na_2_SO_4_and 15 mM HEPES (pH 7.5). Hypotonic low chloride buffer was 67.5 mM sodium-gluconate, 2.5 mM potassium-gluconate, 0.25 mM CaCl_2_, 0.25 mM MgCl_2_, 0.5 mM Na_2_HPO_4_, 0.5 mM Na_2_SO_4_ and 7.5 mM HEPES (pH 7.5).

### Cell culture, transfections and stimulations

HEK293 (human embryonic kidney 293) cells were cultured on 10-cm-diameter dishes in DMEM supplemented with 10% (v/v) fetal bovine serum, 2 mM L-glutamine, 100 U/ml penicillin and 0.1 mg/ml streptomycin. For transfection experiments, each dish of adherent HEK293 cells was transfected with 20 μl of 1 mg/ml polyethylenimine (Polysciences) and 5–10 μg of plasmid DNA as described previously^68^. 36 hours post-transfection cells were stimulated with either control isotonic or hypotonic medium for a period of 30 minutes. HEK-293 cells overexpressing WNK3 (WNK3-WT) and HEK-293 cells expressing WNK3 mutant (WNK3-KD) were cultured in DMEM supplemented with 10% tetracycline free FBS, 10 μg/ml blasticidin, 100 μg/ml hygromycin B, and 5% penicillin-streptomycin. For live cell imaging experiments, 0.2 × 10^6^ cells/well were plated on poly-D-Lysine coated glass coverslips (22 mm × 22 mm) in 6-well plates. KCC3 expression (WT or Mutant) was induced by treatment of cultures with 1 μg/ml doxycycline for 16 h. Cells were lysed in 0.3 ml of ice-cold lysis buffer/dish, lysates were clarified by centrifugation at 4 °C for 15 minutes at 26,000 g, and aliquoted supernatants were frozen in liquid nitrogen and stored at −20 °C. Protein concentrations were determined using the Bradford method. Where noted, cells were treated with the indicated concentrations of the SPAK/OSR1 CCT domain inhibitor STOCK1S-50699 (InterBioScreen Ltd.)^35^.

### Cell volume measurements

Cell volume change was determined using calcein as a marker of intracellular water volume, as described previously^18^. Briefly, cells on coverslips were incubated with 0.5 μM calcein-AM for 30 min at 37 °C. The cells were placed in a heated (37 °C) imaging chamber (Warner Instruments, Hamden, CT) on a Nikon Ti Eclipse inverted epifluorescence microscope equipped with perfect focus, a 40X Super Fluor oil immersion objective lens, and a Princeton Instruments MicroMax CCD camera. Calcein fluorescence was monitored using a FITC filter set (excitation 480 nm, emission 535 nm, Chroma Technology, Rockingham, VT). Images were collected every 60 sec with MetaFluor image-acquisition software (Molecular Devices, Sunnyvale, CA) and regions of interest (~20–30 cells) were selected. Baseline drift resulting from photobleaching and dye leakage was corrected as described^69^. The fluorescence change was plotted as a function of the reciprocal of the relative osmotic pressure and the resulting calibration curve applied to all subsequent experiments as previously described^69^. The HEPES-buffered isotonic solution contained (in mM, pH 7.4): 100 NaCl, 5.4 KCl, 1.3 CaCl_2_, 0.8 MgSO_4_, 20 HEPES, 5.5 glucose, 0.4 NaHC0_3_, and 70 sucrose, adjusted to 310 mOsm using an osmometer (Advanced Instruments, Norwood, MA). Anisosmotic solutions (150, 280 mOsm) were prepared by removal or addition of sucrose to the above solution.

### Immunoblotting and phospho-antibody immunoprecipitation

Cell lysates (15 μg) in SDS sample buffer were subjected to electrophoresis on polyacrylamide gels and transferred to nitrocellulose membranes. The membranes were incubated for 30 min with TTBS containing 5% (w/v) skim milk. The membranes were then immunoblotted overnight at 4 °C in TTBS with 5% skim milk plus the indicated primary antibodies. Sheep antibodies were used at a concentration of 1–2 μg/ml. Incubation with phospho-specific sheep antibodies was in the added presence of 10 μg/ml of the dephosphorylated form of the phosphopeptide antigen used to raise the antibody. The blots were then washed six times with TTBS and incubated for 1 hour at room temperature with secondary HRP-conjugated antibodies diluted 5000-fold in 5% (w/v) skim milk in TTBS. After repeating the washing steps, signals were detected with enhanced chemiluminescence reagent. Immunoblots were developed using a film automatic processor (SRX-101; Konica Minolta Medical) and films were scanned at 600 dpi (PowerLook 1000; UMAX). Figures were generated using Photoshop/Illustrator (Adobe). For phospho-antibody immunoprecipitation, KCC isoforms were immunoprecipitated from indicated cell extracts. 2 mg of the indicated clarified cell extract were mixed with 15 μg of the indicated phospho-specific KCC antibody conjugated to 15 μl of protein-G–Sepharose in the added presence of 20 μg of the dephosphorylated form of the phosphopeptide antigen, and incubated 2 hours at 4 °C with gentle shaking. Immunoprecipitates were washed three times with 1 ml of lysis buffer containing 0.15 M NaCl and twice with 1 ml of buffer A. Bound proteins were eluted with 1x LDS sample buffer.

### Mass spectrometric analysis (MS) analysis

Lysates (5 mg) derived from HEK-293 cells stably expressing wild-type or mutant FLAG epitope-tagged KCC3 were subjected to immunoprecipitation with anti-FLAG antibody covalently conjugated to agarose (5 μl). Immunoprecipitates were washed three times with lysis buffer containing 0.5 M NaCl, followed by two washes with Buffer A. Proteins were eluted from FLAG beads by resuspendion of immunoprecipitates in SDS sample buffer (30 μl). The immunoprecipitates were subjected to electrophoresis on a precast 4–12% gradient gel (Invitrogen) and the protein bands were visualized following Colloidal Blue staining. Proteins in the selected gel bands were reduced and alkylated by the addition of 10 mM DTT, followed by 50 mM iodoacetamide. Identification of proteins was performed by in-gel digestion of the proteins with 5 μg/ml trypsin and subsequent analysis of the tryptic peptides by LC (liquid chromatography)–MS/MS (tandem MS) on a Thermo LTQ-Orbitrap system coupled to a Thermo Easy nano-LC instrument. Excalibur RAW files were converted into peak lists by Raw2msm^70^ and then analysed by Mascot (http://www.matrixscience.com), utilizing the SwissProt human database. Two missed cleavages were permitted; the significance threshold was *P* < 0.05.

### ^86^Rb^+^ uptake assay in ES and HEK293 cells

ES cells were plated in 12-well plates (2.4 cm diameter/well) and the ^86^Rb^+^ uptake assay was performed on cells that were 80% confluent. HEK-293 cells were plated at a confluence of 50–60% in 12-well plates (2.4-cm-diameter per/well) and transfected with wild-type or various mutant forms of full-length flag-tagged human KCCs. Each well of HEK-293 cells was transfected with 2.5 μl of 1 mg/ml polyethylenimine and 1 μg of plasmid DNA. The ^86^Rb^+^-uptake assay was performed on the cells at 36 hours post-transfection. In both cases, culture medium was removed from the wells and replaced with either isotonic or hypotonic medium for 15 min at 37 °C. Cell medium was removed by means of aspiration with a vacuum pump and replaced with stimulating medium containing 1 mM ouabain and 0.1 mM bumetanide, to prevent ^86^Rb^+^ uptake via the NKCC1 cotransporter, for a further 15 min. After this period, the medium was removed and replaced with isotonic medium plus inhibitors containing 2 μCi/ml ^86^Rb^+^ for 10 min at 37 °C. After this incubation period, cells were rapidly washed three times with the respective ice-cold non-radioactive medium. The cells were lysed in 300 μl of ice-cold lysis buffer and ^86^Rb^+^ uptake was quantitated by liquid scintillation counting (PerkinElmer), and was quantified by scintillation counting with transformation of ^86^Rb^+^ uptake counts per minute into flux values (pmoles K^+^/mg protein/min).

### Generation of WNK3 or WNK1 knockout cells using CRISPR/Cas9 gene editing

Analysis of the *PRKWNK3* locus shows that there are 4 transcripts (ENST00000354646, ENST00000375169, ENST00000375159 and ENST00000458404) in this gene. Potential KO CRISPR guide RNAs were subsequently identified using a Sanger Centre CRISPR webtool (http://www.sanger.ac.uk/htgt/wge/find_crisprs). The sequence between exon3 and exon7 in WNK3 gene was replaced with a resistance gene cassette. Cas9/sgRNA mediated indels also contributed to the gene knockout. Three guide RNAs were designed. sgRNA1 (GCTCAGCTTTGGTTAACTTTCGG) was chosen to generate indels in the region of the ATG start codon; an additional G was added to the 5′ end of each guide to maximize expression from the U6 promoter. Complementary oligos were designed and annealed to yield dsDNA inserts with compatible overhangs to BbsI-digested vectors^71^. Guide RNA pairs were cloned into a WT spCas9 and sgRNA expression plasmid. Donor plasmid was constructed by ligating the homologous arm into the TV-B1 vector (Beijing Biocytogen Co. Ltd). HEK293T cells were co-transfected with 1 μg of TV-4G-EB-WNK3 and 3 μg PCS-sgRNA in a 10 cm dish using the Neon Transfection System with Pulse Voltage 1500. Following 24 h recovery and a further 48 h selection with puromycin (1 μg/ml) the transfection was repeated and cells subjected to a further round of puromycin selection to enrich for transfectants. Resistant clones picked with cylinders were analysed for WNK3 depletion by immunoblotting and sequencing. Genomic DNA was isolated for PCR amplification of the region surrounding the exon containing the WNK3 ATG start codon (forward primer WNK3-GT-F: 5′-AGGGCAGAAATACACAAGGAAAGGA-3′; reverse primer PGK-GT-R: 5′-AGAAAGCGAAGGAGCAAAGCTGCTA-3′). The resulting PCR products were subcloned into the holding vector pSC-B (StrataClone Blunt PCR Cloning Kit, Agilent Technologies). Twelve white colonies picked for each clonal line were further confirmed by PCR (forward primer WNK3-MSD-F: 5′-GCCATGTTGGAGGAGTCACAGTAGC-3′; reverse primer WNK3-MSD-R: 5′-TGGCACTATCAGGGTCAACTTACGTC-3′). Isolated plasmid DNAs were Xbal-cut to verify insert size before sequence confirmation with M13F and M13R primers. CRISPR PCR products are heterogeneous due to differences among the targeted alleles. We have found that analysis of >10 heterogeneous post-CRISPR clones per clonal cell line suffices to verify the allelic population. Sequencing of exon 1 PCR fragments from the CRISPR lines revealed a 1859 base-pair deletion (encompassing the start codon) and a 391 base-pair insertion confirming the presence of frameshifting indels and successful KO of the WNK3 loci. Generation of WNK1 knockout cells by CRISPR/Cas9 gene editing was previously described^72^.

### Animals

The SPAK^502A/502A^ knock-in mouse was established and maintained as described in our recent study^47^. The WNK3 knockout (KO) colony was established and maintained as described recently^56^. Kcc1^−/−^Kcc3^−/−^ mouse was established and maintained as described previously^49^. Mice were maintained under specific pathogen-free conditions at the University of Dundee (UK). All animal studies were ethically reviewed and carried out in accordance with Animals (Scientific Procedures) Act 1986, the Policy on the Care, Welfare and Treatment of Animals, regulations set by the University of Dundee and the U.K. Home Office. Animal studies and breeding were approved by the University of Dundee ethical committee and performed under a U.K. Home Office project license.

### Transient focal cerebral ischemia model

Transient focal cerebral ischemia was induced in mice (8–10 weeks old, 25–30 g) by intraluminal occlusion of the left middle cerebral artery (MCA) for 60 min as described previously^56^. Mice were anesthetized with 3% isoflurane in 67%:30% N_2_O/O_2_ until they were unresponsive to the tail pinch test. Animals were then fitted with a nose cone blowing 1.5% isoflurane for anesthesia maintenance. The left common carotid artery was exposed and the occipital artery branches of the external carotid artery were isolated and coagulated. The internal carotid artery was isolated and the extracranial branch was dissected and ligated. A rubber silicon-coated monofilament suture (6–0) was introduced into the internal carotid artery lumen and gently advanced approximately 9–9.5 mm to block the MCA blood flow for 60 min. The rectal temperature was maintained at 37.0 ± 0.5 °C during surgery through a temperature-controlled heating pad. Achievement of ischemia was confirmed by monitoring regional cerebral blood flow (rCBF) in the area of left MCA with a laser Doppler probe as described previously^73^. Briefly, changes in rCBF at the surface of the left cortex were recorded using a blood perfusion monitor (Laserflo BPM2, Vasamedics, Eden Prairie, MN, USA) with a fiber optic probe (0.7 mm in diameter). The tip of the probe was fixed with glue on the skull over the core area supplied by the MCA (2 mm posterior and 6 mm lateral from the bregma). Animals failing to achieve CBF reduction >75% of baseline level or that died after ischemia induction (fewer than 10%) were excluded from further experimentation. The MCA suture was withdrawn to initiate reperfusion. The incision was closed and the mice allowed to recover 30–60 min under a heat lamp to maintain core temperature (36.0–37.0 °C) during the recovery period. After recovery, animals were returned to their cages with free access to food and water.

### Statistical analysis

Data are presented as means ± SEM. Comparison for means between two groups was analyzed by Student t-test (2-tailed). One-way or Two-way repeated measures ANOVA was used to assess statistical significance among multiple group experiments and assays, followed by Tukey’s multiple comparisons test. For all statistical analysis we considered P < 0.05 to be statistically significant. GraphPad Prism (version 7.0, GraphPad Software, Inc., La Jolla, CA) was used for all statistical tests.

S.E.M. values of mean ratios of phospho-protein band intensity (numerator) to total protein band intensity (denominator) were calculated without taking into account the independent s.e.m. values of numerator and denominator inputs (applicable to ratios presented in Figs 2A–C, 3D, 4E and 6B,D). The denominators in these experiments (total protein band intensities) remained unchanged in these experiments with nearly all relative errors <3%, such that changes in ratio were overwhelmingly attributable to changes in numerator (phophoprotein band intensities). The p values for comparisons of these ratios, computed as described above, are indicated in the relevant text and figure legends by *italicized p values*.

All recombinant proteins, DNA constructs, antibodies, generated for this study at the University of Dundee can be requested on our reagents website (https://mrcppureagents.dundee.ac.uk/).

## Additional Information

**How to cite this article**: Zhang, J. *et al*. Functional kinomics establishes a critical node of volume-sensitive cation-Cl^−^ cotransporter regulation in the mammalian brain. *Sci. Rep.* **6**, 35986; doi: 10.1038/srep35986 (2016).

**Publisher’s note:** Springer Nature remains neutral with regard to jurisdictional claims in published maps and institutional affiliations.

## Supplementary Material

Supplementary Information

## Figures and Tables

**Figure 1:** An RNAi screen to identify kinases essential for KCC3 Thr^991^ phosphorylation. (**A**) Characterization of HEK293 cells with doxycycline (dox)-inducible MYC-KCC3 expression used in the RNAi screen. KCC3 wild type (WT) and KCC3 Thr^991^Ala/Thr^1048^Ala protein expression was induced by 0.1 μg/ml doxycycline in the culture medium for 24 hours^19^. Cell lysates were subjected to Western immunoblot (IB) analysis with the indicated antibodies (**B**) Characterization of anti-KCC3 P-Thr^991^ and anti-KCC3 P-Thr^1048^ phospho-specific antibodies. 36 hours post-transfection with the indicated FLAG-tagged constructs, HEK293 cells were treated for 30 min with either isotonic conditions or hypotonic high K^+^ conditions. Total cell extracts were subjected to IB analysis with the indicated antibodies. Mutation of these residues to alanine (Ala^991^ and Ala^1048^) prevented phosphorylation and eliminated the phospho-specific antibody signal at both sites. (**C**) Scheme of the RNAi screen using the human Dharmacon SMARTpool siRNA kinome library to identify essential kinase regulators of KCC3 Thr^991^ phosphorylation. (**D**) Example of results from the primary siRNA screen. Band density of KCC3 P-Thr^991^ from Western blots was quantitated by ImageJ software, and these values were used to calculate the magnitude of KCC3 P-Thr^991^ increase or decrease by comparing to values derived from Firefly (FF) luciferase negative controls. The heat map depicts the average scores for each kinase siRNA pool in the screen that decreased (green) or increased (red) the signal of KCC3 P-Thr^991^ relative to that of the FF siRNA. See Methods for further details. (**E**) Scattered and sorted robust z-scores of kinase hits from the siRNA primary screen. Several siRNA pools led to a significant decrease in the KCC3 P-Thr^991^ signal (>50%, *p* < *0.01* compared to FF siRNA negative control). (**F**) Summary of kinase hits from the secondary siRNA screen. siRNAs targeting primary screen hits were analyzed for their ability to decrease KCC3 P-Thr^991^ without affecting total KCC3 level. The (KCC3 P-Thr^991^)/(total MYC-KCC3) ratio was calculated for each target based on the quantification of immuno-reactive signals in triplicate Western blots, with a value of 100% for FF. Ratios were compared by one-way ANOVA (n = 3, mean ± SEM), with *p* < *0.01* considered statistically significant.

**Figure 2:** Assessment of RNAi screen hits on volume-regulated KCC3 and NKCC1 phosphorylation. (**A**) Assessment of candidate kinase WNK3. We validated secondary siRNA screen hits using cell lines harboring specific knockout (KO) of the target gene of interest to avoid off-target effects of siRNA. WT and WNK3 KO cells^60^ were incubated 30 min in the absence or presence of STOCK1S-50699 (IN), a SPAK conserved carboxy-terminal (CCT) docking domain inhibitor (see Methods). The lysates were immunoprecipitated (IP) and/or immunoblotted (IB) with the indicated antibodies (see also Supplementary Figure 1A,B). The ratio (KCC3 P-Thr^991^)/(total KCC3) ratio was calculated for each kinase KO lysate. Ratios were compared by unpaired t-test (n = 3, mean ± SD). ***p < *0.001*; **p < *0.01*; *p < *0.05*; ns, non-significant. (**B**) Assessment of candidate kinase PDK1. WT and PDK1 KO cells^74^ were treated and analyzed as in (**A**). See also Supplementary Figure 2A,C,D. (**C**) Assessment of candidate kinases AKT1/SGK1. TSC1 or TSC2 KO cells were used as models of down-regulated AKT1 and SGK1 activity^75^, and treated and analyzed as in (**A**). See also Supplementary Figure 2B,C.

**Figure 3:** A screen to identify kinase inhibitors that antagonize KCC3 Thr^991^/Thr^1048^ phosphorylation. (**A**) Results from the primary kinase inhibitor screen. We performed a screen to identify kinase inhibitors that decreased KCC3 P-Thr^991^ using a library of >220 well-characterized, cell-permeable protein kinase inhibitors (see Methods). Dox-induced HEK293-KCC3 WT cells were exposed to 20 μM of kinase inhibitor for 2 hours in 24-well plates. Lysates were harvested, subjected to SDS-PAGE, and Western blot with the indicated antibodies. Quantitative measurement of the KCC3 P-Thr^991^: MYC signal ratio (MYC) was performed as described in Methods. Top hits from the screen are listed below a representative blot from the screen. Drugs showed overlap under several different signaling pathways listed in different colors. (**B**) Results from the secondary kinase inhibitor screen. We tested representative drugs targeting pathways that scored positively in the primary screen at lower concentrations and with decreased incubation times (1 μM for 30 min) to promote inhibitor specificity for the intended target kinase. HEK293 cells expressing N-terminal FLAG epitope tagged KCC3 were treated 30 min with isotonic low Cl^−^ and hypotonic low Cl^−^ conditions, then treated in the same conditions with the indicated inhibitor concentrations for an additional 30 min. (**C**) Concentration-response experiments of STOCK1S-50699 on KCC3 P-Thr^991^/Thr^1048^. HEK293 cells were transfected with DNA construct encoding wild type N-terminal FLAG-tagged KCC3. 36 h post-transfection, cells were exposed 30 min to either control isotonic conditions or hypotonic low Cl^−^ conditions, then treated in the same conditions with STOCK1S-50699 at the indicated concentrations for an additional 30 min. Lysates were and subjected to SDS-PAGE and Western blotting with the indicated antibodies (lower panel). (**D**) Quantitation of immunoblot data from (**C**) presented as ratios of phospho-KCC3/total KCC3. ***p < *0.001*, **p < *0.01*, *p < *0.05*, ns: non-significant.

**Figure 4:** WNK3-SPAK regulates the phosphorylation and function of KCC3. (**A**) ^86^Rb^+^ uptake assays in WNK3 WT and KO ES cells. WT and WNK3 KO cells^60^ were incubated with the indicated isotonic and hypotonic conditions (see Methods) for 30 min in the presence of 1 mM ouabain and 0.1 mM bumetanide. ^86^Rb^+^ uptake proceeded for 10 min and was quantified by scintillation counting. Results are presented as means ± SEM for triplicate samples. ***p < 0.001; **p < 0.01; *p < 0.05, when compared to WT values under the same conditions. (**B**) ^86^Rb^+^ uptake assays in WNK3 and WNK1 KO HEK293 cells. The indicated cells were transfected with constructs encoding a Flag empty vector or the indicated WT or mutant constructs (against KCC3 Thr^991^ and Thr^1048^) of N-terminal FLAG-tagged KCC3. 36 h post-transfection, cells were treated for 30 min with the indicated conditions and ^86^Rb^+^ uptake assays were then carried out in the presence of 1 mM ouabain and 0.1 mM bumetanide and quantitated by scintillation counting. Results are presented as in (**A**). Cell lysates from in parallel experiment were also subjected to immunoblot analysis (Supplementary Figure 4D,E). (**C**) ^86^Rb^+^ uptake assays in the presence of STOCK1S-50699. HEK293 cells were transfected and treated as in (**B**). 10 min ^86^Rb^+^ uptake assays were carried out in the presence of 1 mM ouabain and 0.1 mM bumetanide plus 10 μM of STOCK1S-50699 (indicated in the figure as +IN) and quantitated by scintillation counting. (**D**) HEK293T WT, WNK3 KO and WNK1 KO cells (see Methods) were treated for the indicated times with the indicated conditions. Harvested cell lysates were subjected immunoprecipitation (IP) and/or immunoblot (IB) with the indicated antibodies. (**E**) Graphs show quantitation of Western blot ratios (phospho-KCC3)/(total KCC3) (n = 3, means ± SD). ***p < *0.001*; **p < *0.01*; *p < *0.05*; ns: non-significant (unpaired t-test). Under hypotonic low Cl^−^ conditions, WNK1 KO cells and WNK3 KO cells both exhibited apparently decreased phosphorylation of heterologous KCC3 at Thr^991^ (*p* < *0.001*) and Thr^1048^ (*p* < *0.001*). WNK1 KO HEK293T cells and WNK3 KO HEK293T cells exhibited apparent decreases in phosphorylation of NKCC1 Thr^203^/Thr^207^/Thr^212^, SPAK Ser^373^, and OSR1 Ser^325^ (*p* < *0.05*).

**Figure 5:** Inhibition of WNK3-SPAK signaling prevents acute cell swelling in response to osmotic stress by stimulating KCC3 activity. (**A**) Left panel: Relative change in cell water volume during hypotonic stress in WNK3 WT and WNK3-KD (kinase-dead) cells. Cells were sequentially exposed to isotonic HEPES-MEM (310 mOsm/kg H_2_O), followed by hypotonic HEPES-MEM (150 mOsm/kg H_2_O) to promote cell swelling for 20 min, and then isotonic HEPES-MEM for 5 min. Middle panel: Summary data of cell volume increase. Right panel: Rate constants from the slopes (blue and red lines in left panel) were calculated by fitting a linear regression to the cell water data (relative change) during the initial swelling response (5–7 min). WNK3-KD cells exhibited significantly less swelling in response to hypotonic stress. Data are mean ± SEM, n = 5–6 experiments. *p < 0.05 vs. WT. (**B**) Relative change in cell water after hypotonic swelling in WNK3-WT cells in the presence and absence of STOCK1S-50699. Cells were pre-incubated with 10 μM STOCK1S-50699 for 30 min at 37 degrees C and exposed to osmotic stress as described above in the presence of drug. STOCK1S-50699 prevented cells from swelling in response to acute hypotonic stress. Data are means ± SEM, n = 5–6 experiments. *p < 0.05 vs. WT. (**C**) Relative change in cell water after hypotonic swelling in WNK3-KD cells in the presence and absence of STOCK1S-50699, as described above. Data are means ± SEM, n = 4–5 experiments. No significant difference in either peak change of cell water content or the initial rate of cell swelling was noted with STOCK1S-50699 in WNK3-KD cells. (**D**) Relative change in cell volume in WNK3-WT and WNK3-KD cells in the presence or absence of furosemide. Cells were pre-incubated with 2 mM furosemide for 15 min prior to hypotonic stimulation as described above in the presence of drug. Right panel: Summary data of cell volume increase. The effect of WNK3-KD on decreasing cell swelling is reversed by 2 mM furosemide, revealing a dependence on KCC3 activity. Data are mean ± SEM, n = 3–4 experiments. *p < 0.05.

**Figure 6:** WNK3-SPAK inhibition attenuates the cytotoxic edema of astrocytes and endothelial cells of the blood-brain barrier by decreasing NKCC1/KCC3 phosphorylation. (**A**) Effect of WNK3 knockout on NKCC1 and KCC3 expression and phosphorylation *in vivo*. WT WNK3 and WNK3 KO mice^56^ were subjected to transient middle cerebral artery occlusion (MCAO), a model of ischemic brain swelling^44^. Whole brain homogenates were subjected to immunoprecipitation (IP) and/or immunoblot (IB) with the indicated antibodies. Lysates were immunoblotted in parallel. Molecular masses (kDa) are indicated at the left. (**B**) Bar graphs present the ratio of the phosphorylated target signal to total target intensity (mean+/− SD). *p < *0.05*; **p < *0.01*; ***p < *0.001*. CL: contralateral; IL: ipsilateral. WNK3 KO mice exhibit apparently decreased KCC3 P-Thr^1048^ and NKCC1 P-Thr^203^/Thr^207^/Thr^212^ signals. (**C**) Effect of genetic WNK-SPAK inhibition on NKCC1 and KCC3 expression and phosphorylation *in vivo*. Whole brain homogenates from WT and SPAK CCT L502A knock-in mice^47^ (SPAK^502A/502A^), engineered to mimic WNK-SPAK inhibition by STOCK1S-50699, were subjected to IP and/or IB with the indicated antibodies. Co-immunoprecipitation of KCC3 with SPAK was abrogated in SPAK502A/502A mice. (**D**) Bar graphs summarize ratios of phosphorylated target signal to total target intensity (mean+/− SD). *p < *0.05*; **p < *0.01*; ***p < *0.001*. Similar to WNK3 KO mice, SPAK^502A/502A^ mice exhibit apparently decreased KCC3 P-Thr^1048^ and NKCC1 P-Thr^203^/Thr^207^/Thr^212^ signals. (**E**) Co-immunoprecipitation experiments of WNK3, SPAK, and KCC3 in brain. Whole-brain lysates harvested from WT, KCC1/3 KO, and WNK3 KO mice were immunoprecipitated with the indicated WNK3, SPAK, and KCC3 antibodies, fractionated by SDS-PAGE, and subjected to Western blot analysis with the indicated antibodies. Results are representative of 3 independent experiments. WNK3-SPAK-KCC3 forms a physical complex in mammalian brain. (**F**) Effect of WNK3 KO on the cell volume of peri-infarct reactive astrocytes after MCAO. Representative immunofluorescent images are shown of WNK3 WT (arrows) and WNK3 KO brains (arrowheads) 72 h after MCAO. The soma volume of glial fibrillary acidic protein (GFAP)-positive astrocytes was measured in z-stacks using Imaris software (Version 8.2, Bitplane, Zurich, Switzerland) as described in Methods. Relative to WNK3 WT mice, reactive astrocytes from WNK3 KO mice exhibit significantly reduced cytotoxic edema after MCAO. Values are expressed as Mean ± SEM, n = 3; *p < *0.05* compared to WT. (**G**) Effect of WNK3 KO on blood-brain-barrier (BBB) integrity after MCAO. Representative immunofluorescent images are shown of infiltrated IgG in the brain parenchyma of WNK3 WT and WNK3 KO mice 72 h after MCAO. Bar graph summarizes the results of IgG infiltration. Relative to WNK3 WT mice, WNK3 KO mice exhibit decreased intraparenchymal infiltration IgG after MCAO, indicating less BBB breakdown. Values are expressed as mean ± SEM (n = 5), *p < 0.05 compared to WT.

**Figure 7:** WNK3-SPAK: a “Cl^−^/volume-sensitive kinase” of the cation-Cl^−^ cotransporters and molecular rheostat of cell volume in the mammalian brain. (**A**) A proposed phosphorylation motif in *SLC12A* family NKCC1 and the KCC cotransporters, including KCC3, is shown in a segment of the human KCC1–4 C terminus aligned with a segment of the NKCC1, NCC and NKCC2 N-terminus from human (h) (Revised from ref. 19). The threonine (T) highlighted in yellow indicates a single phosphorylation site that is common to all the transporters. With nearby shared tyrosine (Y) and arginine (R) residues separated by any amino acid residue (X), a candidate *SLC12A* family regulatory phosphorylation motif is suggested. In KCC3, the highlighted Thr in yellow is Thr^991^. Phosphorylation at Thr^212^ in human NKCC1 (Thr^184^ in shark) by WNK1-SPAK kinase signaling is a key event (along with Thr^203^ and Thr^207^) required for NKCC1 activation in conditions that simultaneously promote the inhibitory phosphorylation of KCC3 Thr^991^ 12,28,76. KCC3 Thr^991^ (and homologous sites in other KCCs) and NKCC1 Thr^212^ may be part of a phospho-motif “YXRT” that is important for the coordinated control of NKCCs and the KCCs by the WNK3-SPAK kinase complex (as in **B**). (**B**) Coupling of the WNK3-SPAK kinase complex to NKCC1 and KCC3 could comprise a “molecular rheostat” of cell volume regulation. The WNK3-SPAK kinases may have dual functions as sensors of both cell volume and intracellular [Cl^−^], as well as transducers that communicate changes of these parameters to plasmalemmal ion transport proteins. NKCC1 (“in-flow”) is activated and KCC3 (“out-flow”) is inhibited by WNK3-SPAK-dependent phosphorylation at the indicated sites, leading to regulatory volume increase (RVI, in blue to left of rheostat) that mediates net accumulation of intracellular solute – as would occur in response to prior cell shrinkage. In the opposite scenario, NKCC1 is inhibited and KCC3 is activated by WNK3-SPAK inhibition and by activation of protein phosphatases, leading to decreased NKCC1/KCC3 phosphorylation. The resulting regulatory volume decrease (RVD, in red to right of rheostat) regulatory volume decrease (RVI, in blue to left of rheostat) that mediates net reduction of intracellular solute – as would occur in response to cell swelling. Therefore, the WNK3-SPAK complex might function as a “sensor-transducer” of cell volume perturbations that, via a physical and functional coupling to NKCC1 and KCC3, comprises a molecular rheostat of cell volume.

**Table 1:** A kinase trapping-Orbitrap mass spectroscopy screen to identify kinase regulators of KCC3.

		Target	Mascot Protein Score	Peptide Match (unique peptides)	Sequence Coverage
Phosphorylated KCC3	Basic Lysate	PRMT5 (O14744)	192	5	10%
		MASTL (Q96GX5)	105	3	5%
		TLK2 (Q86UE8)	79	3	5%
	Hypotonic Lysate	STK39 (Q9UEW8)	63	2	7%
		PRMT5 (O14744)	85	3	6%
		MTOR (P42345)	83	2	1%
Dephosphorylated KCC3	Basic Lysate	STK39 (Q9UEW8)	161	2	7%
		TLK2 (Q86UE8)	86	3	5%
		CALM1 (P62158)	49	2	35%
		MTOR (P42345)	115	5	2%
		PRMT5 (O14744)	256	6	12%
	Hypotonic Lysate	STK39 (Q9UEW8)	91	3	9%
		PRMT5 (O14744)	84	3	5%
		MTOR (P42345)	98	4	2%
		PGK1 (P00558)	151	2	6%

Accession numbers are from SwissProt. Data only contains peptides whose ion score in Mascot was greater than 26 and hence with p < 0.05.
